# Increased Anterior Pelvic Angle Characterizes the Gait of Children with Attention Deficit/Hyperactivity Disorder (ADHD)

**DOI:** 10.1371/journal.pone.0170096

**Published:** 2017-01-18

**Authors:** Hiroaki Naruse, Takashi X. Fujisawa, Chiho Yatsuga, Masafumi Kubota, Hideaki Matsuo, Shinichiro Takiguchi, Seiichiro Shimada, Yuto Imai, Michio Hiratani, Hirotaka Kosaka, Akemi Tomoda

**Affiliations:** 1 Division of Developmental Higher Brain Functions, United Graduate School of Child Development, University of Fukui, Eiheiji-cho, Yoshida-gun, Fukui, Japan; 2 Division of Physical Therapy and Rehabilitation, University of Fukui Hospital, Eiheiji-cho, Yoshida-gun, Fukui, Japan; 3 Research Center for Child Mental Development, University of Fukui, Eiheiji-cho, Yoshida-gun, Fukui, Japan; 4 National Hospital Organization Hizen Psychiatric Center, Kanzaki-gun, Saga, Japan; 5 Department of Child and Adolescent Psychological Medicine, University of Fukui Hospital, Eiheiji-cho, Yoshida-gun, Fukui, Japan; 6 Hiratani Clinic for Developmental Disorders of Children, Kitayotsui, Fukui City, Fukui, Japan; Chiba Daigaku, JAPAN

## Abstract

**Background:**

Children with attention deficit/hyperactivity disorder (ADHD) frequently have motor problems. Previous studies have reported that the characteristic gait in children with ADHD is immature and that subjects demonstrate higher levels of variability in gait characteristics for the lower extremities than healthy controls. However, little is known about body movement during gait in children with ADHD. The purpose of this study was to identify the characteristic body movements associated with ADHD symptoms in children with ADHD.

**Methods:**

Using a three-dimensional motion analysis system, we compared gait variables in boys with ADHD (n = 19; mean age, 9.58 years) and boys with typical development (TD) (n = 21; mean age, 10.71 years) to determine the specific gait characteristics related to ADHD symptoms. We assessed spatiotemporal gait variables (i.e. speed, stride length, and cadence), and kinematic gait variables (i.e. angle of pelvis, hip, knee, and ankle) to measure body movement when walking at a self-selected pace.

**Results:**

In comparison with the TD group, the ADHD group demonstrated significantly higher values in cadence (*t* = 3.33, *p* = 0.002) and anterior pelvic angle (*t* = 3.08, *p* = 0.004). In multiple regression analysis, anterior pelvic angle was associated with the ADHD rating scale hyperactive/impulsive scores (*β* = 0.62, *t* = 2.58, *p* = 0.025), but not other psychiatric symptoms in the ADHD group.

**Conclusions:**

Our results suggest that anterior pelvic angle represents a specific gait variable related to ADHD symptoms. Our kinematic findings could have potential implications for evaluating the body movement in boys with ADHD.

## Introduction

Attention deficit hyperactivity disorder (ADHD) is the most prevalent childhood onset neurodevelopmental disorder, affecting 7.2% of school-age children [1]. ADHD is characterized by age-inappropriate level of inattention, hyperactivity, and impulsivity that are present prior to age 12 years of age [2]. Additionally, up to 50% of children with ADHD demonstrate a subnormal level of motor performance in their age group [3–6]. Previous studies have reported that poor coordination and impairments in fine and gross motor function are caused by difficulty in directing attention and by display of impulsive behavior [7, 8]. To date, motor function, including gait function, has been clinically assessed as a neurological soft sign in children with ADHD [9]. Gait function is one of the fundamental motor skills requiring both attention and executive function [7, 10]. From MRI studies, children with ADHD have a reduction in volume of the cerebellum [11] and dysfunction of the circuits involving basal ganglia [12]. These brain regions have a role in regulating the balance during gait [13, 14] and gait abnormalities have been reported in this population. However, there are few reports based on objective measurements using instrumented gait analysis techniques.

Previous studies of gait in children with ADHD have mainly focused on the differences of gait variables in children with ADHD [15], or age-dependent change in gait that bring children with ADHD closer to typically developed controls [16]. Step length in children with ADHD has shown great variability, which becomes much more pronounced during dual tasking, and is reduced to levels approaching those of control subjects after initiating medication [15]. In addition, a tendency toward a higher value for step frequency has been reported, which becomes more pronounced during tasks requiring regulation of gait speed [17]. In contrast, when walking on the treadmill, no differences in step length and frequency were reported [18]. In brief, the gait characteristics common in children with ADHD are a faster pace and higher variability with each step during free gait. Furthermore, these gait characteristics appear to be most prominent when attention is redirected to another task during gait. To date, previous studies have only measured these characteristics spatiotemporally, although there have been a few studies measuring body movement during gait. One study reported measurements of body movement during a continuous performance seated task, providing objective measurements using a motion analysis system to study factors associated with hyperactive behavior, which subsequently provided insight into the motor activity of children with ADHD [19].

Three-dimensional (3D) motion analysis, which uses an infrared camera to assess body movement in terms of gait kinematics, has been helpful for investigating and understanding body movement to determine disease-specific gait characteristics [20]. For pediatric populations, gait characteristics involving body movement have been identified in children with autism spectrum disorders (ASD) [21] and developmental coordination disorder (DCD) [22]. For instance, stride length and duration variation, lack of motor smoothness, and head and trunk posture abnormalities have been reported in children with ASD [23, 24]. Moreover, children with DCD reportedly have shorter stride length, higher cadence, reduced range of motion in the lower extremities, flexion of the upper body, and increased complexity and variation in lower limb movement patterns [25]. As described before, body movements during gait have not been clarified, although spatiotemporal gait characteristics have been identified in children with ADHD.

The aim of this study was to identify the kinematic gait characteristics of children with ADHD to measure the body movement of gait quantitatively. Furthermore, to determine the ADHD-specific gait characteristics, we sought to assess further whether alterations in gait variables are associated with psychiatric symptom measurements. We predicted that the severity of ADHD is related to the kinematic gait variables that have significant differences between children with ADHD and children with typical development.

## Methods

### Ethics statement

The protocol of this study was approved by the Ethics Committee of the University of Fukui (Assurance No. 20130066). After reading a complete description of the study, all participants and their parents provided written informed consent for participation. The experimental protocol was conducted in accordance with the Declaration of Helsinki.

### Participants

This study examined 19 boys with ADHD aged 7–12 years [9.58 ± 1.84 years (mean ± S.D.)]. Each child had been referred to the Department of Child and Adolescent Psychological Medicine, University of Fukui Hospital. Diagnosis was made following DSM-5 [2] and DSM-IV ADHD items taken from the DSM- IV modified Schedule for Affective Disorders and Schizophrenia for School Age Children—Epidemiologic Version by experienced child and adolescent psychiatrists (C. Y., S. T., H. K., and A.T.). Children were categorized as ADHD combined type (n = 11) and ADHD inattentive type (n = 8) using ADHD rating scale Japanese version (ADHD-RS). Participants attended the gait laboratory in Fukui University Hospital where testing took place from October 2013 to August 2014. Most ADHD children in this study (15/19) were taking medication such as methylphenidate (MPH) 0.7–2.1 mg/kg per day or atomoxetine (ATX) 0.1–0.9 mg/kg per day. For patients taking medication, the washout duration for MPH was at least 24 hours, and for ATX it was at least 1 week. Furthermore, there were no children meeting the criteria of ASD or DCD. The control group consisted of 21 boys, typically developed children aged 7–14 years [10.71 ± 2.05 years (mean ± S.D.)] who were recruited for this study from the community in Fukui Prefecture, and matched for age and handedness. Intelligence was evaluated using the Wechsler Intelligence Scale for Children Fourth Edition or Third Edition (WISC-IV or WISC-III) [26, 27]. Exclusion criteria for all patients were any history of orthopedic disorder within the prior 6 months, past diagnosis of any psychiatric disorder, head trauma with loss of consciousness, epilepsy, presence or absence of significant fetal exposure to alcohol or drugs as disclosed by their parents, perinatal or neonatal complications, neurological disorders, premature birth (gestation ≤36 weeks), and diagnosis of any bipolar, psychotic, obsessive—compulsive, or tic disorder at any point in their lifetime.

### Questionnaires

To evaluate the severity of ADHD symptoms, we used ADHD-RS, an 18-item questionnaire [28]. Each item was scored by frequency of occurrence (i.e., if the patient “never” presented the symptom, it is coded as 0; if “occasionally”, 1; “often”, 2; and “always”, 3. Total scores could range from 0 to 54, with higher scores indicating more severe ADHD symptoms. Several previous studies reported the presence of comorbid disorders such as ASD or DCD in many children with ADHD [29] who had an alteration of gait [20–25]. Therefore, we assessed for ASD and DCD traits to identify the specificity related to ADHD symptoms. The Autism Spectrum Quotient Japanese Children’s Version (AQ) [30], a 50-item questionnaire, was completed by a parent to evaluate ASD traits, such as social skills, attention switching, attention to detail, communication, and imagination. The Movement Assessment Battery for Children Second Edition (M-ABC2) [31] (Pearson Ltd., London, UK), which has eight subtests, was used to assess DCD traits, such as manual dexterity, ball skills, and static and dynamic balance.

### Gait analysis measurement

We measured gait variables (spatiotemporal and kinematic gait variables) by using a 3D motion analysis system (VICON-MX) that included ten T10 cameras (Vicon Motion Systems Ltd., Oxford, UK) and four synchronized force plates (Advanced Mechanical Technology Inc., Watertown, MA, USA) placed in the middle of a 10-meter walkway (Fig 1). We placed two cones at each end of the walkway. All cameras and force plates were calibrated before data collection. The sampling rate was set at 100 Hz for cameras and force plates.

**Fig 1:** Three-dimensional motion analysis system. The system is comprised of 10 strobe cameras mounted from the ceiling and four force plates placed in the middle of the walkway. The white circles represent 14 mm reflective markers according to the Plug-in-Gait marker set.

Height and weight were measured prior to gait assessment to control for body size differences, and spatiotemporal variables were normalized for each trait in accordance with the method described by Hof [32]. The 14 mm retro-reflective markers were placed on anatomical landmarks (front and back of the head, 7^th^ cervical vertebrae, 10^th^ thoracic vertebrae, clavicle, sternum, the middle of right scapula, shoulder, elbow, wrist, anterior superior iliac spine, posterior superior iliac spine, shank, knee, shin, ankle, heel, and toe) according to the Plug-in-Gait marker set. Participants were instructed to walk with bare feet to the cone at their own pace. All participants conducted a few warm-up trials to acclimatize to the gait laboratory setting before placing makers.

### Data processing

All trials in which the force plates were hit were checked visually using Vicon NEXUS motion capture software (Vicon Motion Systems Ltd., Oxford, UK). Error trials, such as ones in which markers fell off or no impact was made on the force plate, were excluded from further analysis. Marker trajectory was reconstructed and filtered using the Woltring filtering routine with Vicon NEXUS. The gait cycle started when one foot touched the floor and ended when that same foot touched the floor again. Gait variables were normalized as a percentage of the gait cycle using Polygon 3 (Vicon Motion Systems Ltd., Oxford, UK).

The assessed spatiotemporal variables were walking speed (m/s), stride length (m), and cadence (steps/min). The kinematic variables consisted of joint angle (degrees) in the sagittal plane for pelvis (Fig 2), hip, knee, and ankle. Peak values in each kinematic variable were extracted. The averages of five trials and right-and-left data were calculated for each participant to maintain the reliability of data from the 3D motion analysis system [33].

**Fig 2:** Schema for pelvic angle in sagittal angle during gait. A shows the pelvic angle. B shows the pelvic angle during gait. Ant: anterior; post: posterior.

### Statistical analysis

Demographic data and gait variables were tested using independent *t* test and clinical symptoms were tested using ANCOVA with age and FISQ as covariates. To examine the correlation between ADHD symptoms based on ADHD-RS scores, and gait variables demonstrating significant differences for both groups, partial correlation coefficients were calculated with FSIQ as a covariate. Additionally, gait variables in children are multifactorial, with contributions from developmental indices (i.e. age and cognitive function) [20, 34] and neurodevelopmental symptoms (i.e. ASD traits or DCD traits) [21–25]. Therefore, to investigate the substantial contribution of ADHD traits to gait characteristics for other variables (age, FSIQ, ASD, and/or DCD traits), we used standard multiple regressions by forced entry method and investigated their relationship. To test our hypothesis that psychiatric symptom measurements could significantly predict gait variables, we performed a multiple regression analysis using psychiatric symptom measures showing significant between-group differences as independent variables, and the gait variables showing significant between-group differences as dependent variables. The statistical threshold was set at *p* < 0.05 and used the Bonferroni adjustment for multiple comparisons. All analyses were conducted using the Statistical Package for the Social Sciences 20 software (SPSS Inc., Chicago, IL, USA).

## Results

Demographic and clinical characteristics for the study participants are listed in Table 1. In comparison with the TD group, the ADHD group scored significantly lower on the FSIQ (*t* = 2.70, *p* = 0.011). Significant differences were found in the measures of severity of ADHD symptoms (ADHD-RS total score, *F* [1, 36] = 101.18, *p* < 0.001; Inattentive score, *F* [1, 36] = 79.92, *p* < 0.001; Hyperactive/Impulsive score, *F* [1, 36] = 42.08, *p* < 0.001), ASD traits (AQ total; *F* [1, 36] = 18.95, *p* < 0.001), and DCD traits (M-ABC2 total; *F* [1, 36] = 3.76, *p* = 0.060) between the two groups.

**Table 1:** Demographic and clinical characteristics of ADHD and TD groups.

Variables	Group			
	ADHD	TD	Statistics	*p*-value
*Demographic characteristics*				
Subject (n)	19	21		
Age (years)^†^	9.58 (1.84)	10.71 (2.05)	1.85	0.073
Handedness (n, L/R)	3/16	3/18	0.01	0.894
Height (m) ^†^	1.37 (0.13)	1.46 (0.14)	1.97	0.056
Weight (kg) ^†^	32.79 (8.82)	37.68 (12.61)	1.42	0.163
FSIQ^a,^ ^†^	98.05 (13.16)	108.71 (11.68)	2.70	0.011*
*Clinical characteristics*^‡^				
ADHD-RS				
Total	28.79 (9.08)	2.90 (3.11)	101.18	<0.001**
Inattentive	17.84 (5.80)	2.14 (2.39)	79.92	<0.001**
Hyperactive /Impulsive	11.37 (6.08)	0.76 (1.18)	42.08	<0.001**
AQ total	20.28 (5.06)	12.10 (4.12)	18.95	<0.001**
M-ABC2 total	9.74 (2.42)	12.48 (2.44)	3.76	0.060

Data are presented as mean (SD). a: FSIQ data were based on the WISC-IV (n = 37) and WISC-III (n = 3). Data were not available for one subject because of a missing value for AQ (ADHD, 1 subject). FSIQ = Full Scale Intelligence Quotient; AQ = The Autism Spectrum Quotient-Children's Version; M-ABC2 = Movement Assessment Battery for Children Second edition.

^†^ Group difference was tested by independent t-test.

^‡^ Group difference was tested by ANVOCA with age and FSIQ as covariate.

The statistical threshold is set at * p < 0.05 and ** p < 0.01.

Gait variables are shown in Table 2. Between-group comparisons for spatiotemporal and kinematic gait variables were assessed by independent *t* test. In comparison with the TD group, the ADHD group showed significantly higher cadence in spatiotemporal variables (*t* = 3.33, *p* = 0.002), and also showed significantly higher anterior pelvic angle (*t* = 3.08, *p* = 0.004). Normalization of the data according to Hof [32] did not alter any of the findings for between-group differences in gait variables. Therefore, we adopted the data before normalization for statistical analysis.

**Table 2:** Differences in gait variables between ADHD and TD groups.

Variables	Group			
	ADHD (n = 19)	TD (n = 21)	Statistics	*p*-value
*Spatiotemporal variables*				
Walking Speed (m/s)	1.21 (0.61)	1.19 (0.18)	0.61	0.546
Stride length (m)	1.17 (0.15)	1.21 (0.18)	-0.91	0.369
Cadence (steps/min)	125.26 (6.72)	117.40 (8.19)	3.33	0.002**
*Kinematic variables* (degree)				
Anterior pelvic angle	13.13 (5.24)	8.59 (4.36)	3.08	0.004**
Hip flexion angle	34.04 (6.87)	28.72 (5.97)	2.65	0.012
Hip extension angle	11.93 (5.42)	15.56 (6.57)	2.05	0.047
Knee flexion angle	54.60 (3.93)	54.55 (6.48)	0.11	0.915
Knee extension angle	1.30 (3.57)	2.79 (3.84)	1.20	0.237
Ankle dorsal-flexion angle	15.28 (4.01)	15.97 (5.40)	-0.44	0.662
Ankle Plantar-flexion angle	14.79 (5.51)	14.72 (6.27)	0.10	0.919

Data are shown as mean (±SD). Group differences were tested by independent *t* test. The statistical threshold is set at ** *p* < 0.005 using the Bonferroni adjustment for multiple comparisons.

To assess the relationship between gait variables and ADHD symptoms, we explored the correlation between the gait variables and ADHD-RS scores beginning with the inter-correlation of the gait variables. There was no significant correlation between the kinematic variables and cadence as a spatiotemporal variable (*r* = 0.17, *p* = 0.287). Therefore, we adopted pelvic angle and cadence as the representative gait variables for the following correlation analysis with ADHD symptoms. Since we observed a significant difference in FSIQ between groups, we calculated partial correlation coefficients between these gait variables and ADHD symptoms, controlling for FSIQ. As shown in Fig 3A, we observed significant partial correlation coefficients between cadence and ADHD-RS total scores in the entire group (ADHD and TD) (*r* = 0.38, *p* = 0.018), whereas there were no significant correlations between these variables in each group separately (ADHD: *r* = -0.10, *p* = 0.690; TD: *r* = 0.03, *p* = 0.912). In contrast, as shown in Fig 3B, we observed significant partial correlation coefficients between pelvic angle and ADHD-RS total score in the ADHD group (*r* = 0.54, *p* = 0.021) as well as in the whole group (*r* = 0.65, *p* < 0.001), whereas no significant correlation was observed in the TD group (*r* = 0.24, *p* = 0.306). These results suggest the possibility that pelvic angle is specifically associated with the severity of ADHD symptoms.

**Fig 3:** Partial correlation analysis of gait variables and ADHD rating scale. These show correlation between ADHD-RS and cadence (A), or pelvic angle (B) with FSIQ as covariate. Blue circle and solid line: TD group; Red circle and solid line: ADHD group; Black dotted line: all subjects.

Next, we determined the core set of variables to develop an explanatory model of gait. We then performed multiple regression analyses to further characterize the relationship between psychiatric symptom measures and gait variables such as cadence and pelvic angle. For cadence, as shown in Table 3, a higher cadence was associated with a decreased age (*β* = -0.34, *t* = -2.08, *p* = 0.046) in all subjects, although there were no associations with any psychiatric symptoms. For pelvic angle, however, a higher anterior pelvic angle was associated with an increased ADHD-RS score in all subjects. As indicated in Table 4, our analysis showed that the severity of ADHD symptom measures, based on ADHD-RS hyperactive/impulsive score (*β* = 0.52, *t* = 2.40, *p* = 0.023), and cognitive ability, based on FSIQ (*β* = 0.35, *t* = 2.16, *p* = 0.038), were significant predictors for anterior pelvic angle in all subjects, and explained approximately 33% of the variance in the pelvic angle (adjusted *R*^2^ = 0.33, *F* [6,32] = 4.15, *p* = 0.003). However, anterior pelvic angle had no association with AQ (*β* = 0.14, *t* = 0.82, *p* = 0.419) or M-ABC2 (*β* = -0.15, *t* = -0.91, *p* = 0.368). In the ADHD group, anterior pelvic angle also had an association with ADHD-RS hyperactive/impulsive score (*β* = 0.62, *t* = 2.58, *p* = 0.025), and explained approximately 21% of the variance in the pelvic angle (adjusted *R*^2^ = 0.21, *F* [6,11] = 1.76, *p* = 0.197). In the TD group, anterior pelvic angle had an association with FSIQ (*β* = 0.59, *t* = 2.27, *p* = 0.040).

**Table 3:** Regression model statistics and coefficients of variables for cadence.

	All (n = 40)		ADHD (n = 19)		TD (n = 21)	
Independent	β	*t-value*	β	*t-value*	β	*t-value*
ADHD-RS						
Inattentive	0.165	0.60	-0.46	-1.12	0.02	0.05
Hyperactive/impulsive	0.136	0.56	0.02	0.07	-0.06	-0.18
Age	-0.34*	-2.08	-0.15	-0.45	-0.43	-1.55
FSIQ	0.06	0.31	0.09	0.31	0.07	0.234
AQ	-0.07	-0.36	-0.50	-1.50	-0.14	-0.46
M-ABC2	-0.19	-1.07	-0.25	-0.71	-0.17	-0.64
Adjusted *R*^2^	0.18		-0.06		-0.21	

Standardized regression coefficients (β), *t* values, and *R*^*2*^ are reported. The corrected statistical threshold is set at * *p* < 0.05. For the analysis, one subject data was not available due to a missing value in AQ (ADHD, 1 subject).

**Table 4:** Regression model statistics and coefficients of variables for anterior pelvic angle.

	All (n = 40)		ADHD (n = 19)		TD (n = 21)	
Independent	β	*t-value*	β	*t-value*	β	*t*-value
ADHD-RS						
Inattentive	0.06	0.23	0.02	0.05	0.44	1.67
Hyperactive/impulsive	0.52*	2.40	0.62*	2.58	-0.47	-1.52
Age	0.03	0.21	0.09	0.32	-0.09	-0.35
FSIQ	0.35*	2.16	0.32	1.25	0.59*	2.27
AQ	0.14	0.82	0.15	0.52	0.27	0.99
M-ABC2	-0.15	-0.91	-0.23	-0.76	-0.18	-0.75
Adjusted *R*^2^	0.33**		0.21		-0.07	

Standardized regression coefficients (β), *t* values, and *R*^*2*^ are reported. The corrected statistical threshold is set at * * *p* < 0.01 and * *p* < 0.05. For the analysis, one subject data was not available due to a missing value in AQ (ADHD, 1 subject).

## Discussion

The purpose of the present study was to determine whether spatiotemporal and kinematic gait variables differ between controls and children with ADHD by using a 3D motion analysis system. Our results demonstrated that children with ADHD exhibit higher values for cadence and anterior pelvic angle compared to healthy controls, and that pelvic angle had a significant positive correlation with the severity of ADHD symptoms. These results suggest that children with ADHD have the characteristics of a high frequency gait cycle and an increased anterior pelvic angle. Furthermore, in multiple regression analysis, anterior pelvic angle was associated with the severity of ADHD symptoms, whereas there was no association with ASD or DCD symptoms in children with ADHD. Additionally, the variable of cadence showed no association with any psychiatric traits. These findings suggest that increased anterior pelvic angle during gait is a specific variable of ADHD symptoms.

As expected, cadence, a spatiotemporal variable, had a positive correlation with ADHD symptoms in all subjects. A recent study reported that children with ADHD walked faster and with a higher cadence and that ADHD symptoms were associated with increased cadence in the “fast walking condition” [17]. Although we could not determine the underlying mechanism for higher cadence in children with ADHD, one possible explanation is that difficulties in timing regulation may be attributed to cerebellar dysfunction [35], which is one area consistently implicated as a neural basis for ADHD [36]. Nevertheless, it is noteworthy that many previous studies have reported gait abnormalities in spatiotemporal variables, including higher cadence, in children with other neurodevelopmental disorders, such as ASD or DCD [21, 22]. As demonstrated by the results of the multiple regression analysis in the present study, we did not observe any significant association between cadence and ADHD symptoms or other psychiatric traits of ASD and DCD, suggesting that cadence may not be a variable specifically related to ADHD pathogenesis. Instead, spatiotemporal gait variables, including cadence, may reflect heterogeneous clinical conditions between ADHD and other neurodevelopmental disorders, making it difficult to determine whether cadence is a critical gait characteristic related to ADHD symptoms.

Curiously, in the present investigation we found a positive association between pelvic angle as a kinematic gait variable and ADHD symptoms. Why pelvic angle might be associated with ADHD is an interesting question. Pelvic movement is essential as an inherent mechanism of postural control in normal children [37] and has often been observed clinically to estimate the biomechanics of different gait patterns [38]. An increased anterior pelvic angle is necessary to move the center of gravity forward in order to walk efficiently [39]. Specifically, pelvic angle is determined by the muscle strength or stiffness around the pelvis needed to maintain upright posture, which is regulated by the basal ganglia and/or cerebellar vermis [14, 40]. Increased anterior tilt angle has been observed in infants, implicating an immature neuromuscular system [37, 41]. A meta-analysis of functional magnetic resonance imaging (fMRI) studies in children with ADHD revealed a neurological delay in basal ganglia development [42]. In children with ADHD, meta-analysis suggested that deregulation of front-basal ganglia-parietal network may cause the deficit of attention and inhibition [12]. These brain networks, known as the motor loop, involve the basal ganglia and have a role in generating the gait pattern and control for muscle tone to regulate gait and posture. Moreover, meta-analysis of structural imaging reported a volume reduction of the cerebellar vermis [43], which has been related to inattentive symptoms [44] and verbal working memory performance in children with ADHD. The cerebellum has a role of maintaining equilibrium during gait. Another previous study reported that step variability decreases with age. Together, these studies suggest that immature gait is related to delayed brain development [15]. Although we have discussed this finding in terms of a potential cause and effect mechanism, it must be emphasized that our evidence only supports an association.

Moreover, as suggested by multiple regression analysis, we have observed that anterior pelvic angle shows an association with the severity of ADHD symptoms, although it shows no association with ASD or DCD symptoms, suggesting that pelvic angle may be one of the candidates for gait-specific variables in ADHD. To the best of our knowledge, the present study is the first to clarify the association between kinematic gait variables and the severity of ADHD symptoms.

There were several limitations of this study. The first major limitation is the small sample size in this study. The cleanliness of the sample (all drug-naive, very narrow age range, no other form of ASD or DCD traits, matched socio-economic status, past histories of sports activities) might have compensated for that shortcoming, at least in part, by reducing error variance. To generalize our results, studies involving a larger number of participants must be conducted to compare with children with ASD or DCD. Second, this study used a cross-sectional design that precludes identification of causal links between ADHD and gait variables. Longitudinal studies must be conducted to investigate how gait variable differences associated with ADHD change in response to treatment programs aimed at diminishing signs of ADHD.

In conclusion, increased anterior pelvic angle was associated with increased severity of ADHD symptoms. These preliminary findings could have potential implications for our understanding of gait control related to ADHD and a possible contribution for evaluating the body movement in boys with ADHD. Combining 3D motion analysis for body movement with neurophysiological indicators of brain activity should prove fruitful in further elucidating the mechanisms underlying motor control in children with ADHD.

## Supporting Information

S1 Dataset The demographic, psychology assessments and gait data. (XLSX)
